# Body composition and mortality in a cohort study of Chinese patients with hypertrophic cardiomyopathy

**DOI:** 10.3389/fcvm.2023.988274

**Published:** 2023-03-15

**Authors:** Ke Zhou, Jie Xiang, Guo-yong Li, Xiao-bo Pu, Li Zhang

**Affiliations:** ^1^ Cardiology Department, Affiliated Minda Hospital of Hubei Minzu University, Enshi, China; ^2^ Cardiac Pacing and Electrophysiological Department, The First Affiliated Hospital of Xinjiang Medical University, Urumqi, China; ^3^ Xinjiang Key Laboratory of Cardiac Electrophysiology and Cardiac Remodeling, The First Affiliated Hospital of Xinjiang Medical University, Urumqi, China; ^4^ Cardiology Department, West China Hospital, Sichuan University, Chengdu, China

**Keywords:** hypertrophic cardiomyopathy, obesity paradox, body mass index, LEAN MASS, body fat

## Abstract

**Objective:**

To analyse the characteristics and mortality of hypertrophic cardiomyopathy (HCM) patients with different body compositions.

**Methods:**

In this study, 530 consecutive patients with HCM at West China Hospital were studied from November 2008 to May 2016. An equation based on body mass index (BMI) was used to obtain the Percent body fat (BF) and lean mass index (LMI). Patients were divided into five sex-specific BMI, BF and LMI quintiles.

**Results:**

The average BMI, BF and LMI were 23.1 ± 3.2 kg/m^2^, 28.1 ± 7.3% and 16.5 ± 2.2 kg/m^2^, respectively. Patients with higher BMI or BF were older and had more symptoms and adverse cardiovascular conditions; those with higher LMI were younger and had less coronary artery disease and lower serum NT-proBNP and creatine. BF correlated positively with resting left ventricular (LV) outflow tract gradient, mitral regurgitation (MR) degree and left atrial diameter but was inversely associated with septal wall thickness (SWT), posterior wall thickness (PWT), LV mass, and E/A ratio; LMI was positively correlated with SWT, LV end diastolic volume and LV mass but was negatively associated with MR degree.48 all-cause deaths occurred during a median follow-up of 33.8 months. Reversed J-shape associations of BMI and LMI with mortality were observed. A lower BMI or LMI was significantly associated with high mortality, especially for low-moderate BMI and LMI. No significant difference in mortality was found across BF quintiles.

**Conclusions:**

The associations of BMI, BF and LMI with baseline characteristics and cardiac remodelling are different in HCM patients. In Chinese HCM patients, low BMI and LMI predicted mortality but not BF.

## Introduction

Hypertrophic cardiomyopathy (HCM) is the most common inherited heart disorder with heterogeneity in its natural history. Although HCM-causing mutations are believed to be the main prognostic factor of HCM patients, a gene-based model is still unable to predict outcomes (1). In fact, even classically inherited diseases can be modified by demographic features, physiological challenges and comorbid conditions. Therefore, understanding the relationship between environmental modulators and outcomes can help manage patients with HCM.

Obesity has become a major health concern as a result of the change in modern lifestyles. The population with obesity is more vulnerable to cardiovascular disease. However, in the context of chronic diseases, including chronic heart failure (2), chronic obstructive pulmonary disease (3), and stroke (4), higher body mass index (BMI) closely associated with lower mortality, presenting an “obesity paradox”. With respect to HCM, it has been reported that obesity in adolescence predicts a higher occurrence rate of HCM in midlife (5). However, it is unclear whether there is an obesity paradox in patients with HCM.

BMI, an index universally applied to measure obesity, has been questioned under the background of the obesity paradox in cardiovascular disease (6). Fat mass and lean mass are included in body composition, and BMI does not differentiate between these components. Having a high BMI does not necessarily mean that you have a higher body fat (BF), but may indicate that you have a higher lean mass. Thus, the paradox, resulting from the apply of an inaccurate surrogate for obesity, may be a misleading finding. For example, a recent study from our group showed that among coronary artery disease patients with mild renal insufficiency, there was no association between fat mass and mortality risk, but an inverse association between lean mass and mortality risk (7). However, data on the effect of body composition on survival in HCM patients are limited. In the present study, the objective was to investigate the relationship between body composition and mortality in a Chinese cohort with HCM.

## Methods

### Subjects

The data of this study were obtained from the hypertrophic cardiomyopathy database of West China Hospital. The database includes data from consecutive patients diagnosed with HCM at West China Hospital of Sichuan University from November 2008 to May 2016, and the collected data includes demographic, clinical, laboratory and treatment data. Patients with the following conditions will be excluded: (1) patients with malignant tumors, (2) patients with severe aortic valve disease and (3) patients with end-stage renal failure. All patients have been informed consent, so that their medical records for research purposes. The study got the West China Hospital of Sichuan University Ethics Committee approval.

### Echocardiographic evaluation

All patients were assessed by echocardiography as recommended by the American Society of Echocardiography (8). Two-dimensional echocardiography was used to diagnose HCM based on a left ventricular (LV) wall thickness ≥ 15 mm in adults who did not have any cardiac or systemic etiology that can cause such hypertrophy (9, 10). Resting left ventricular outflow tract (LVOT) obstruction was determined by apical five-chamber view with a peak outflow gradient ≥ 30 mmHg at rest (11). The continuity equation method was used to analyze the regurgitant jet area, vena contracta width and regurgitation quantitation, and then the mitral regurgitation (MR) was divided into no, mild, moderate and severe regurgitation (12). With the following formula to determine LV mass: LV mass = 0.8{1.04[(LV external end-diastolic diameter (LVEDD) + PWTd + SWT)^3^ − (LVEDD)^3^]} + 0.6 g.

### Body composition assessment

Using standard methods, nurses measured the patients' height and weight, and calculated BMI by dividing the weight (kg) by the square of the height (m^2^). The Clínica Universidad de Navarr—Body Adiposity Estimator (CUN-BAE) equation was applied to estimate percentage BF: BF = −44.988 + (0.503 × age) + (10.689 × sex) + (3.172 × BMI) − (0.026 × BMI^2^) + (0.181 × BMI × sex) − (0.02 × BMI × age) − (0.005 × BMI^2^ × sex) + (0.00021 × BMI^2^ ×age), where sex is replaced by 0 for males and 1 for females (13).This formula has been verified in previous study (14). The formula (1 − BF%) × BMI kg/m^2^ was applied to calculate the lean mass index (15). Because there were no reports of reference value in the Chinese population, study patients were divided into five groups based on the quintiles of sex-specific BMI, LMI and BF.

### Baseline data collection and laboratory measurement

The baseline anthropometric data were obtained from electronic medical records. The medical history (hypertension, diabetes mellitus, coronary artery disease, stroke and dyslipidaemia), symptoms of HCM, smoking history, and family history of sudden cardiac death were obtained from hospital records and collected by trained research investigators. Cardiologists assess the risk of sudden cardiac death (SCD) according to the HCM Risk-SCD tool (16). Venous blood samples were collected in tubes containing ethylene diamine tetraacetic acid (EDTA) and analysed at the Department of Laboratory Medicine, West China Hospital, accredited by the College of American Pathology.

### Events and follow-up

During follow-up, the primary event recorded was all-cause mortality and the secondary event was cardiovascular mortality. Patients themselves and/or their family members were contacted by telephone or through outpatient visits for follow-up information. Most of the patients visited outpatient appointments every 1–6 months. All the data were consistent with the hospital records.

### Patient and public involvement

It was inappropriate or impossible to involve patients or the public in the design, or implementation, or reporting, or dissemination plans of our study.

### Statistical analysis

Continuous variables with a normally distributed distribution are presented as the mean ± standard deviation, while non-normally distributed variables are presented as the median (interquartile range). Categorical variables are represented as counts (percentages). The *χ*^2^ test or Fisher's exact test was applied to compare categorical variables. Data were compared using one-way analysis of variance if they followed a normal distribution; or else, the data were compared using the Kruskal-Wallis test. Single correlations between body composition and echocardiographic characteristics were evaluated using Pearson's correlation test when the values were normally distributed; otherwise, they were analysed using Spearman's rank correlation test. To determine the association between body composition and outcomes, survival across body composition categories was plotted in Kaplan-Meier curves and compared using the log-rank test. Then, multivariate Cox proportional hazard analyses were applied to identify the independent effects of baseline body composition characteristics on time until death. Possible confounding factors of age, sex and medical history (diabetes mellitus, hypertension, atrial fibrillation, coronary artery disease and family history of SCD) were adjusted; septal wall thickness (SWT); LVOT obstruction; LV wall thickness > 30 mm; LV ejection fraction (LVEF); treatment with β blockers, non-dihydropyridine calcium channel blockers, angiotensin-converting enzyme inhibitors or angiotensin-receptor blockers; and alcohol septal ablation. The method described by Grambsch and Therneau was used to assess the assumption of proportional hazards (17). Restricted spline regression analyses, using four knots, were performed to test the potential non-linear relationship of body composition with all-cause mortality. The fitted spline model for all-cause mortality vs. each body composition characteristic was then plotted on the log-hazards scale, with confidence intervals overlaid. All statistical analyses were conducted using Stata/MP 13.0. We considered a two-sided *P* value <0.05 to be statistically significant.

## Results

530 patients with complete BMI data from the West China Hospital Hypertrophic Cardiomyopathy database were included in the present study. The average age of these patients was 54.5 ± 16.4 years, and 54.2% of the enrolled patients were male. The average BMI, BF and LMI were 23.1 ± 3.2 kg/m^2^, 28.1 ± 7.3% and 16.5 ± 2.2 kg/m^2^, respectively. The distributions of the patients' baseline data across BMI, LMI and BF quintiles are showed in Tables 1–3, respectively. In general, patients with higher BMI or BF were older; had a higher frequency of chest pain symptoms, more comorbidities (hypertension, diabetes, stroke or coronary artery disease), and a higher level of serum creatine; and were more likely to be on statins. More patients with lower BF were classified as having a moderate-high risk of SCD. In contrast, patients with higher LMI had a significantly lower age. A lower proportion of patients with higher LMI had a history of coronary artery disease. Lower serum levels of creatine and NT-proBNP were found among patients with higher LMI. Loop diuretics were prescribed less often in patients with higher LMI.

**Table 1:** Baseline characteristics to sex-specific BMI quintiles.

Characteristics	Total	Sex-specific BMI strata					
		Quintile1	Quintile2	Quintile3	Quintile4	Quintile5	*p*
Number of patients	530	107	107	106	107	103	
Ages, years	54.5 (16.4)	48.2 (20)	56.5 (14.5)	55.6 (16.6)	56.4 (14.5)	56.1 (14.4)	***<0*** *.* ***001***
Male, *n* (%)	287 (54.2)	58 (54.2)	58 (54.2)	58 (54.7)	57 (53.3)	56 (54.4)	1.000
LMI, kg/m^2^ (SD)	16.5 (2.2)	15.1 (2.0)	16.0 (1.8)	16.5 (1.9)	16.9 (2.0)	18.1 (2.2)	***<0***.***001***
BMI, kg/m^2^ (SD)	23.1 (3.2)	19.2 (1.9)	21.7 (1.0)	22.9 (0.9)	24.2 (1.1)	27.5 (2.6)	***<0***.***001***
BF, % (SD)	28.1 (7.3)	21.4 (6.9)	26.7 (5.4)	28.3 (6.0)	30.3 (5.7)	34.3 (5.8)	***<0***.***001***
**Symptoms, *n* (%)**							
Chest pain	152 (28.7)	21 (19.6)	35 (32.7)	37 (34.9)	28 (26.2)	31 (30.1)	0.108
Dyspnea	223 (42.1)	47 (43.9)	47 (43.9)	43 (40.6)	43 (40.2)	43 (41.8)	0.967
Syncope	167 (31.5)	33 (33.8)	30 (28.0)	31 (29.3)	37 (34.6)	6 (35.0)	0.753
Hypertension, *n* (%)	182 (34.3)	22 (20.6)	36 (33.6)	44 (41.5)	37 (34.6)	43 (41.8)	***0***.***007***
Diabetes mellitus, *n* (%)	42 (7.9)	5 (4.7)	9 (8.4)	10 (9.4)	5 (4.7)	13 (12.6)	0.160
Coronary artery disease, *n* (%)	92 (17.4)	13 (12.2)	19 (17.8)	25 (23.6)	20 (18.7)	15 (14.6)	0.232
Hyperlipidemia, *n* (%)	33 (6.2)	6 (5.6)	2 (1.9)	7 (6.6)	6 (5.6)	12 (11.6)	0.065
Stroke, *n* (%)	17 (3.2)	1 (0.9)	2 (1.9)	5 (4.7)	8 (7.5)	1 (1.0)	***0***.***025***
Family history of SCD, *n* (%)	7 (1.3)	3 (2.8)	3 (2.8)	0	1 (0.9)	0	0.163
NYHA class III-IV, *n* (%)	202 (38.1)	40 (37.4)	36 (33.6)	41 (38.7)	36 (33.6)	49 (47.6)	0.218
NT-proBNP, pg/ml (IQR)	1,013 (334–2,788)	1,131 (367–3,013)	943 (256–3,241)	934 (408–2,671)	1,218 (376–2,857)	629 (235–2,374)	0.233
Creatine, µmol/L	80 (66.6–93)	79 (64.7–94.6)	80 (67–93.5)	77.6 (64.5–89)	81.5 (69–98)	80.3 (67–91.8)	0.401
HCM risk-SCD, *n* (%)							0.675
Low risk*	373 (70.4)	73 (68.2)	76 (71.0)	76 (71.7)	72 (67.3)	76 (73.8)	
Moderate risk*	115 (21.7)	22 (20.6)	23 (21.5)	21 (19.8)	25 (3.4)	24 (23.3)	
High risk*	42 (7.9)	2 (11.2)	8 (7.5)	9 (8.5)	10 (9.4)	3 (2.9)	
**ECG features, *n* (%)**							
Atrial fibrillation	71 (13.4)	12 (11.2)	17 (15.9)	16 (15.1)	13 (12.2)	13 (12.6)	0.832
Bundle branch block	54 (10.2)	17 (15.9)	9 (8.4)	8 (7.6)	11 (10.3)	9 (8.8)	0.266
NSVT	92 (17.4)	16 (15.0)	15 (14.0)	18 (17.0)	21 (19.6)	22 (21.4)	0.591
SVT	8 (1.5)	1 (0.9)	1 (0.9)	4 (3.8)	1 (0.9)	1 (1.0)	0.334
**Treatment strategies**							
Alcohol septal ablation	42 (7.9)	7 (.5)	7 (6.5)	12 (11.3)	13 (12.2)	3 (2.9)	0.078
Surgical septal myectomy	7 (1.3)	1 (0.93)	2 (1.9)	0	3 (2.8)	4 (1.0)	0.450
Biventricular pacemakers	21 (4.0)	3 (2.8)	8 (7.5)	3 (2.8)	4 (3.7)	3 (2.9)	0.340
ICD implantation	26 (4.9)	4 (3.7)	8 (7.5)	3 (2.8)	5 (4.7)	6 (5.8)	0.557
**Medicines at discharge**							
*β* blokers	395 (74.5)	77 (72.0)	80 (74.8)	79 (74.5)	77 (72.0)	82 (79.6)	0.709
Calcium channel blockers	26 (4.9)	6 (5.6)	6 (5.6)	10 (9.4)	3 (2.8)	1 (1.0)	0.054
ACEI/ARB	18 (3.4)	7 (6.5)	4 (3.7)	2 (1.9)	3 (2.8)	2 (1.9)	0.311
Loop diuretics	123 (23.2)	28 (26.2)	25 (23.4)	25 (23.6)	24 (22.4)	21 (20.4)	0.905
Statins	114 (21.5)	10 (9.4)	20 (18.7)	28 (26.4)	24 (22.4)	32 (31.1)	***0***.***002***
Amiodarone	28 (5.3)	5 (4.7)	5 (4.7)	7 (6.6)	5 (4.7)	6 (5.8)	0.955
Warfarin	42 (7.9)	12 (11.2)	8 (7.5)	9 (8.5)	6 (5.6)	7 (6.8)	0.621

ACEI, angiotensin-converting enzyme inhibitors; ARB, angiotensin receptor bloker; BMI, body mass index; BF, body fat; ECG, electrocardiograph; LMI, lean mass index; SCD, sudden cardiac death; SD, standard deviation. Bold indicates the significantly statistical difference.

Low risk*: HCM risk-SCD < 4 points; Moderate risk*: 4 points ≤HCM risk-SCD < 6 points; High risk*: HCM risk-SCD ≥ 6 points.

**Table 3:** Baseline characteristics to sex-specific LMI quintiles.

Characteristics	Total	Sex-specific LMI strata					
		Quintile1	Quintile2	Quintile3	Quintile4	Quintile5	*p*
Number of patients	530	107	106	106	106	105	
Ages, years (SD)	54.5 (16.4)	62.8 (16.5)	57.9 (15.5)	54.9 (14.2)	50 (15.8)	47.0 (15.2)	***<0*** *.* ***001***
Male, *n* (%)	287 (54.2)	58 (54.2)	57 (53.8)	58 (54.7)	57 (53.8)	57 (54.3)	1
LMI, kg/m^2^ (SD)	16.5 (2.2)	14.8 (1.9)	15.9 (1.7)	16.5 (1.8)	17.1 (2.0)	18.2 (2.2)	***<0***.***001***
BMI, kg/m^2^ (SD)	23.1 (3.2)	19.8 (2.2)	21.7 (1.6)	23.0 (1.4)	24.0 (2.0)	27.0 (3.0)	***<0***.***001***
BF, % (SD)	28.1 (7.3)	24.9 (7.9)	26.8 (6.6)	28.0 (7.1)	28.7 (6.3)	32.3 (6.6)	***<0***.***001***
**Symptoms, *n* (%)**							
Chest pain	152 (28.7)	28 (26.2)	31 (29.3)	33 (31.1)	33 (31.1)	27 (25.7)	0.840
Dyspnea	223 (42.1)	51 (47.7)	42 (39.6)	44 (41.5)	44 (41.5)	42 (40)	0.764
Syncope	167 (31.5)	34 (31.8)	23 (21.7)	39 (36.8)	33 (31.3)	38 (36.2)	0.127
Hypertension, *n* (%)	182 (34.3)	38 (35.5)	36 (34.0)	44 (41.5)	31 (29.3)	33 (31.4)	0.392
Diabetes mellitus, *n* (%)	42 (7.9)	9 (8.4)	9 (8.5)	7 (6.6)	8 (7.6)	9 (8.6)	0.981
Coronary artery disease, *n* (%)	92 (17.4)	26 (24.3)	18 (17.0)	25 (23.6)	13 (12.3)	10 (9.5)	***0***.***012***
Hyperlipidemia, *n* (%)	33 (6.2)	4 (3.7)	5 (4.7)	7 (6.6)	6 (5.7)	11 (10.5)	0.300
Stroke *n* (%)	17 (3.2)	3 (2.8)	3 (2.8)	8 (7.6)	1 (0.9)	2 (1.9)	0.065
Family history of SCD, *n* (%)	7 (1.3)	0	2 (1.9)	3 (2.8)	1 (0.9)	1 (1.0)	0.438
NYHA class III-IV, *n* (%)	202 (38.1)	47 (43.9)	31 (29.3)	39 (36.8)	40 (37.7)	45 (42.9)	0.188
NT-proBNP, pg/ml (IQR)	1,013 (334–2,788)	1,237 (517–5,379)	768 (256–2,450)	1,229 (390–2,863)	1,223.5 (376–2,583)	630 (213–1,938)	***0***.***004***
Creatine, µmol/L	80 (66.6–93)	84.0 (69.4–100.4)	78.5 (62–88)	81.3 (70.5–98)	77.7 (62–92.6)	77.2 (65–90)	***0***.***019***
HCM risk-SCD, *n* (%)							0.300
Low risk*	373 (70.4)	83 (77.6)	82 (77.4)	72 (67.9)	67 (63.2)	69 (65.7)	
Moderate risk*	115 (21.7)	15 (14.0)	15 (14.2)	21 (19.8)	26 (24.5)	22 (21.0)	
High risk*	42 (7.9)	9 (8.4)	9 (8.5)	13 (12.3)	13 (12.3)	14 (13.3)	
**ECG features, *n* (%)**							
Atrial fibrillation	71 (13.4)	19 (17.8)	11 (10.4)	15 (14.2)	16 (15.1)	10 (9.5)	0.372
Bundle branch block	54 (10.2)	13 (12.2)	11 (10.4)	9 (8.5)	13 (12.3)	8 (7.6)	0.728
NSVT	92 (17.4)	16 (15.0)	18 (17.0)	16 (15.1)	20 (18.9)	22 (21.0)	0.748
SVT	8 (1.5)	2 (1.9)	0	3 (2.8)	2 (1.9)	1 (1.0)	0.512
**Treatment strategies**							
Alcohol septal ablation	42 (7.9)	9 (8.4)	6 (5.7)	11 (10.4)	13 (12.3)	3 (2.9)	0.089
Surgical septal myectomy	7 (1.3)	1 (0.9)	1 (0.9)	2 (1.9)	2 (1.9)	1 (1.0)	0.929
Biventricular pacemakers	21 (4.0)	6 (5.6)	3 (2.8)	6 (5.7)	2 (1.9)	4 (3.8)	0.537
ICD implantation	26 (4.9)	2 (1.9)	5 (4.7)	7 (6.6)	7 (6.6)	5 (4.8)	0.487
**Medicines at discharge**							
β blokers	395 (74.5)	74 (69.2)	74 (69.2)	79 (74.5)	87 (82.1)	81 (77.1)	0.170
Calcium channel blockers	26 (4.9)	6 (5.6)	9 (8.5)	5 (4.7)	4 (3.8)	2 (1.9)	0.252
ACEI/ARB	18 (3.4)	5 (4.7)	4 (3.8)	4 (3.8)	4 (3.8)	1 (1.0)	0.630
Loop diuretics	123 (23.2)	28 (26.2)	26 (24.5)	34 (32.1)	21 (19.8)	14 (13.3)	***0***.***019***
Statins	114 (21.5)	25 (23.4)	20 (18.9)	27 (25.5)	19 (17.9)	23 (21.9)	0.652
Amiodarone	28 (5.3)	7 (6.5)	3 (2.8)	4 (3.8)	7 (6.6)	7 (6.7)	0.580
Warfarin	42 (7.9)	14 (13.1)	7 (6.6)	8 (7.6)	9 (8.5)	4 (3.8)	0.155

Low risk*: HCM risk-SCD < 4 points; Moderate risk*: 4 points ≤HCM risk-SCD < 6 points; High risk*: HCM risk-SCD ≥ 6 points.

Bold indicates the significantly statistical difference.

We further explored the potential correlations between body composition and various echocardiographic data (Table 4). BMI was positively correlated with LVEDV but inversely correlated with the E/A ratio. BF was positively associated with the resting LVOT gradient, MR degree and LA diameter but was negatively associated with SWT, posterior wall thickness (PWT), LV mass, and E/A ratio. LMI was positively correlated with SWT, LVEDV and LV mass but was negatively associated with MR degree. No correlation was observed between LVEF and the three body composition measurements.

**Table 4:** Relation of BMI, LMI or BF to echocardiographic characteristics.

	BMI		LMI		BF	
	*r*	*P* value	*r*	*P* value	*r*	*P* value
Resting LVOT gradient (mmHg)	0.035	0.424	−0.064	0.142	0.129	**0**.**003**
Mitral regurgitation degree	−0.010	0.826	−0.138	**0**.**002**	0.180	**<0**.**001**
SWT (mm)	0.035	0.428	0.121	**0**.**005**	−0.141	**0**.**001**
PWT (mm)	−0.024	0.580	0.039	0.366	−0.097	**0**.**026**
LV mass (g)	0.132	**0**.**002**	0.203	**<0**.**001**	−0.099	**0**.**023**
LVEF (mm)	−0.002	0.973	0.016	0.722	−0.030	0.487
LVEDV (ml)	0.218	**<0**.**001**	0.228	**<0**.**001**	−0.010	0.819
LA diameter (mm)	0.070	0.107	−0.034	0.436	0.136	**0**.**002**
E/A ratio	−0.097	**0**.**026**	0.015	0.737	−0.158	**<0**.**001**

LA, left atrium; LVEDV, left ventricular end diastolic volume; LVEF, left ventricular ejection fraction; LVOT, left ventricular outflow tract; PWT, posterior wall thickness; SWT, septal wall thickness. Bold indicates variables significantly correlated with the corresponding body compositions.

Over a median follow-up of 33.8 months (interquartile range, 14.8–58.3 months; maximum follow-up, 107 months), a total of 48 [rate 2.74/100 person-year, 95% confidence interval (CI) 2.07–3.64] deaths occurred, and of those deaths, 31 (rate 1.77/100 person-year, 95% CI 1.25–2.51) were ascribed to cardiovascular causes. Kaplan-Meier plots suggested that the risk of all-cause and cardiovascular mortality was higher in the low BMI group (Figures 1A,B). Similar results were also observed in the low LMI group (*P* for all-cause mortality < 0.001 and *P* for cardiovascular mortality = 0.012, Figures 1C,D). However, no significant difference in mortality was found across the BF groups (*P* for all-cause mortality = 0.545 and *P* for cardiovascular mortality = 0.097, Figures 1E,F).

**Figure 1:** Kaplan-Meier plots according to the quintiles of body composition: (**A,B**) for BMI; (**C,D**) for LMI and (**E,F**) for BF.

The univariate and multivariate HRs for all-cause and cardiovascular mortality by body composition variables are displayed in Supplementary Figure S1. Lower BMI and LMI were associated with higher all-cause mortality. Even after multifactorial correction, BMI (quintile 1: reference; quintile 2: HR 0.31, 95% CI 0.12–0.78; quintile 3: HR 0.60, 95% CI 0.28–1.30; quintile 4: HR 0.33, 95% CI 0.13–0.82; quintile 5: HR 0.37, 85% 0.16–0.90) or LMI (quintile 1: reference; quintile 2: HR 0.21, 95% CI 0.08–0.59; quintile 3: HR 0.37, 95% CI 0.16–0.88; quintile 4: 0.35, 95% CI 0.14–0.87; quintile 5: 0.28, 95% CI 0.10–0.76) were inversely associated with the risk of all-cause mortality (Figure 2A). However, no significant association between BF and mortality could be observed. Similarly, the univariate and multivariate Cox analyses showed that BMI and LMI, but not BF, were inversely relevant to cardiovascular deaths (Figure 2B).

**Figure 2:** Hrs and 95% CIs for all-cause (**A**) and cardiovascular mortality (**B**) associated with different quintiles of body composition. There was no significant violation of the proportional hazard assumption (all-cause death: *P* = 0.36, 0.16 and 0.46 for BMI-, LMI- and BF-containing models, respectively; cardiovascular death: *P* = 0.66, 0.59 and 0.73 for BMI-, LMI- and BF-containing models, respectively).

Spline regression curves demonstrating the multivariable-adjusted HRs of BMI, LMI and BF for risk of death are presented in Figure 3. Figure 3A illustrates a reversed J-shape curve, with an inflexion point occurring at BMI ≤ 23 kg/m^2^, such that a higher BMI was independently correlated with a lower risk of death (Figure 3A). The risk of all-cause mortality was relatively flat when BMI was greater than 23 kg/m^2^. With respect to LMI, the risk of death decreased in a linear fashion until approximately 18 kg/m^2^ of LMI and then started to decrease slowly afterwards (Figure 3B). However, Figure 2C shows an overall U-shaped relationship between BF and all-cause mortality, with the inflexion point at BF = 32%.

**Figure 3:** Splines of the multivariate associations between BMI (**A**), LMI (**B**) or BF (**C**) and all-cause mortality. Adjusted for age; sex; medical history (diabetes mellitus, hypertension, atrial fibrillation, coronary artery disease and family history of SCD); SWT; LVOT obstruction; left ventricular wall thickness > 30 mm; left ventricular ejection fraction; treatment with β blockers, non-dihydropyridine calcium channel blockers, angiotensin-converting enzyme inhibitors or angiotensin-receptor blockers; and alcohol septal ablation. The two dotted lines show the 95% CIs.

## Discussion

In this cohort study of 530 Chinese HCM patients, we used a validated anthropometric prediction equation to examine the association of BF and LMI with all-cause and cardiovascular mortality. We found that mortality was inversely related to BMI, especially among normal weight (BMI ≤ 22 kg/m^2^) HCM patients. The inverse relationship of LMI with mortality seemed to be stronger until approximately 18 kg/m^2^ of LMI. However, BF was not significantly associated with mortality in HCM patients.

Obesity is emerging as a public health problem and a well-known risk factor for cardiovascular disease. Recently, a Sweden nationwide registry-based prospective cohort study showed that obesity in adolescence resulted in an increased risk of HCM in midlife (5). Moreover, Olivotto et al. reported that obesity may contribute to more rapid clinical progression and worsening of heart failure symptoms in HCM patients (18). In agreement with these findings, Larsen et al. suggested that in patients with HCM, increasing BMI was associated with a higher prevalence of dyspnoea and poorer exercise capacity. However, few studies to date have addressed the effect of obesity on mortality in patients with HCM. Our data demonstrated that the frequency of HCM-related symptoms did not differ across BMI groups, but when BMI was less than 23 kg/m^2^, higher BMI predicted a lower risk of death, which seems to be contrary to the above reports. Notably, the U- or reversed J-shape relationship between BMI and outcomes of HCM patients has been documented in both Meghji et al.'s study and the present study. Thus, considering the striking distinction of BMI between Caucasian (mean BMI 30 kg/m^2^) and Chinese (23.1 kg/m^2^) studies, our data may reflect the exclusive relationship between BMI and outcomes in the Chinese HCM population who have relatively low BMI levels.

The obesity paradox has been documented in patients with coronary artery disease, chronic heart failure and several chronic vascular diseases, but it remains controversial. One of the arguments against the obesity paradox focused on the defect of BMI in measuring body composition (lean mass and fat mass). In fact, Oreoponlous et al. showed that BMI, as a surrogate for obesity, had a better relationship with lean mass than BF. BMI-measured obesity is sometimes associated with excess muscle rather than fat (6). Higher BF reflects lower physical activity, hyperinsulinaemia, and more risk factors, while higher LMI may reflect a healthy metabolic state. Thus, people with the same BMI may have entirely different cardiovascular risk profiles. As expected, in our study, patients with higher BF were concomitant with clustered cardiovascular conditions, such as hypertension, diabetes mellitus, coronary artery disease and higher prescriptions of statins (Table 2). Conversely, higher LMI was associated with relatively benign cardiovascular profiles involving a lower frequency of coronary artery disease and diuretic use and lower levels of serum NT-proBNP and creatine (Table 3).

**Table 2:** Baseline characteristics to sex-specific BF quintiles.

Characteristics	Total	Sex-specific BF strata					
		Quintile1	Quintile2	Quintile3	Quintile4	Quintile5	*p*
Number of patients	530	107	106	106	106	105	
Ages, years (SD)	54.5 (16.4)	37.8 (16.1)	50.8 (12.7)	56.9 (11.8)	63.6 (12.0)	63.9 (13.3)	***<0*** *.* ***001***
Male, *n* (%)	287 (54.2)	49 (45.8)	49 (46.2)	48 (45.3)	49 (46.2)	48 (45.7)	1
LMI, kg/m^2^ (SD)	16.5 (2.2)	15.8 (2.0)	16.2 (2.1)	16.4 (2.0)	16.5 (2.1)	17.7 (2.4)	***<0***.***001***
BMI, kg/m^2^ (SD)	23.1 (3.2)	19.8 (2.2)	21.9 (1.8)	22.9 (1.6)	23.8 (1.6)	27.2 (2.9)	***<0***.***001***
BF, % (SD)	28.1 (7.3)	20.5 (6.1)	26.2 (5.2)	28.5 (5.2)	30.8 (5.5)	34.9 (5.6)	***<0***.***001***
**Symptoms, *n* (%)**							
Chest pain	152 (28.7)	18 (16.8)	30 (28.3)	38 (35.9)	35 (33.0)	31 (29.5)	***0***.***026***
Dyspnea	223 (42.1)	45 (42.1)	42 (39.6)	51 (48.1)	46 (43.4)	39 (37.1)	0.563
Syncope	167 (31.5)	32 (29.9)	35 (33.0)	31 (29.3)	33 (31.1)	36 (34.3)	0.928
Hypertension, *n* (%)	182 (34.3)	11 (10.3)	33 (31.1)	31 (29.3)	52 (49.1)	55 (52.4)	***<0***.***001***
Diabetes mellitus, *n* (%)	42 (7.9)	4 (3.7)	6 (5.7)	8 (7.6)	6 (5.7)	18 (17.1)	***0***.***003***
Coronary artery disease, *n* (%)	92 (17.4)	3 (2.8)	18 (17.0)	22 (20.8)	29 (27.4)	20 (19.1)	***<0***.***001***
Hyperlipidemia, *n* (%)	33 (6.2)	5 (4.7)	3 (2.8)	5 (4.7)	10 (9.4)	10 (9.5)	0.148
Stroke *n* (%)	17 (3.2)	0	3 (2.8)	4 (3.8)	5 (4.7)	5 (4.8)	0.258
Family history of SCD, *n* (%)	7 (1.3)	5 (4.7)	1 (0.9)	1 (0.9)	0	0	***0***.***015***
NYHA class III-IV, *n* (%)	202 (38.1)	38 (35.5)	31 (29.3)	43 (40.6)	42 (39.6)	48 (45.7)	0.148
NT-proBNP, pg/ml (IQR)	1,013 (334–2,788)	1,131 (270–2,717)	785 (359–2,760)	1,053 (327–2,368)	1,050.5 (374–3,221)	982 (283–2,771)	0.931
Creatine, µmol/L	80 (66.6–93)	77 (64.5–89)	78 (66–92.8)	77.2 (65–93.2)	79.4 (67–92)	85 (71.1–98)	***0***.***021***
HCM risk-SCD, *n* (%)							***0***.***004***
Low risk*	373 (70.4)	61 (57.0)	70 (60.0)	76 (71.7)	83 (78.3)	83 (79.1)	
Moderate risk*	115 (21.7)	27 (25.2)	28 (26.4)	16 (15.1)	14 (13.2)	14 (13.3)	
High risk*	42 (7.9)	19 (17.8)	8 (7.6)	14 (13.2)	9 (8.5)	8 (7.6)	
**ECG features, *n* (%)**							
Atrial fibrillation	71 (13.4)	12 (11.2)	13 (12.3)	14 (13.2)	15 (14.2)	17 (16.2)	0.858
Bundle branch block	54 (10.2)	12 (11.2)	14 (13.2)	13 (12.3)	6 (5.7)	9 (8.6)	0.360
NSVT	92 (17.4)	11 (10.3)	15 (14.2)	23 (21.7)	22 (20.8)	21 (20)	0.123
SVT	8 (1.5)	0	3 (2.8)	2 (1.9)	3 (2.8)	0	0.212
**Treatment strategies**							
Alcohol septal ablation	42 (7.9)	7 (6.5)	10 (9.4)	11 (10.4)	12 (11.3)	2 (1.90)	0.079
Surgical septal myectomy	7 (1.3)	2 (1.9)	1 (0.9)	2 (1.9)	1 (0.9)	1 (1.0)	0.932
Biventricular pacemakers	21 (4.0)	3 (2.8)	6 (5.7)	4 (3.8)	3 (3.8)	5 (4.8)	0.786
ICD implantation	26 (4.9)	4 (3.7)	9 (8.5)	5 (4.7)	3 (2.8)	5 (4.8)	0.377
**Medicines at discharge**							
β blokers	395 (74.5)	79 (73.8)	77 (72.6)	76 (71.7)	87 (82.1)	76 (72.4)	0.391
Calcium channel blockers	26 (4.9)	4 (3.7)	5 (4.7)	7 (6.6)	7 (6.6)	3 (2.9)	0.631
ACEI/ARB	18 (3.4)	7 (6.5)	3 (2.8)	3 (2.8)	1 (0.9)	4 (3.8)	0.246
Loop diuretics	123 (23.2)	27 (25.2)	20 (18.9)	18 (17.0)	28 (26.4)	30 (28.6)	0.201
Statins	114 (21.5)	5 (4.7)	18 (17.0)	27 (25.5)	27 (25.5)	37 (35.2)	***<0***.***001***
Amiodarone	28 (5.3)	7 (6.5)	5 (4.7)	4 (3.8)	7 (6.6)	5 (4.8)	0.859
Warfarin	42 (7.9)	8 (7.5)	9 (8.5)	8 (7.6)	10 (9.4)	7 (6.7)	0.957

Low risk*: HCM risk-SCD < 4 points; Moderate risk*: 4 points ≤HCM risk-SCD < 6 points; High risk*: HCM risk-SCD ≥ 6 points.

Bold indicates the significantly statistical difference.

Obesity has been shown to result in abnormal cardiac remodelling and function mediated by fat-derived inflammatory cytokines. Olivotto et al. demonstrated that obesity indexed by BMI was associated with increased LV mass and LA diameter, LVEDD and greater LVOT obstruction (15). When considering body composition, we found that higher BF, but not LMI, was associated with diastolic dysfunction and more severe LVOT obstruction, which can be seen from the positive association between BF and LA diameter, MR degree and resting LVOT gradient (Table 4). The increased levels of inflammatory factors and hyperinsulinaemia that usually occur in the presence of increased BF might induce myocardial fibrosis, thereby decreasing ventricular compliance (19). Moreover, our data indicated that LMI appears to be associated with eccentric hypertrophy in HCM patients, which can be seen from the positive correlation between LMI and LVEDV and LV mass. These findings in the context of HCM were similar to those in the general population. Previous studies suggested that athletes with greater lean mass have higher LV mass and LVEDV (20). In fact, an increase in LV mass and LVEDV in patients with high LMI may be understood as a result of an increased circulating blood volume and cardiac output necessary to supply the metabolic demand of lean mass (21). Additionally, genetic influences in regard to HCM may concomitantly affect skeletal muscle. However, even though we observed that individuals with higher LMI have greater LV mass, Miyaji et al. showed that the baseline LV mass was not associated with the clinical outcomes of HCM patients (22).

As far as we know, this is the first study to investigate the relationship between body composition and the mortality of HCM patients. Our data added a new insight that the reversed J-shaped relationship between BMI and morality in HCM patients can be explained by a combination of the association of LMI and BF with mortality. The decreased mortality associated with high BMI within the range of less than 23 kg/m^2^ could be attributed to the low risk of death associated with high lean mass. The stabilized association between BMI and mortality in the higher BMI range (>24 kg/m^2^) was likely due to the counteracting of the opposite influence of BF and LMI on mortality. In fact, the prognostic value of LMI has been documented in a broader population. In a prospective study of an Asian population, Han et al. suggested that higher LMI was associated with better survival; whereas, BF was not associated with mortality (23). Kokkinos et al. suggested that a high mortality rate related with low BMI levels was observed only in patients without high fitness, indicating that the insufficiency of lean mass might be partly responsible for the obesity paradox in individuals with low BMI levels (24). Therefore, our study suggested that more attention should be paid to nutritional supplements in the management of HCM patients, with the hope of increasing their lean mass.

There are some limitations in our research that should be noted. Firstly, although this study looked at the association between body composition and mortality, BF and lean mass were obtained from formulas and not directly measured. Therefore, direct measurement of lean mass and BF using methods such as dual-energy x-ray absorption and bioelectrical impedance requires further investigation. However, in terms of clinical application, the direct measurement of BF and lean mass is unpractical due to its cost. The CUN-BAE equation was obtained by analyzing a large population and subsequently validated in several other studies. In a sense, the assessment of lean mass derived from BMI *via* the CUN-BAE equation can be easier to accept by clinicians. Secondly, this is a retrospective observational study that was conducted in a single tertiary referral centre, with inherent biases compared to real-world studies. Third, the study recruited only Chinese HCM patients with a mean BMI of 23.1 kg/m^2^. Therefore, the extrapolation of these results to other race/ethnicities, especially Caucasians who have much higher BMIs, must be performed cautiously.

## Conclusion

In a cohort of the Chinese population with HCM, we provided evidence showing that when BMI is divided into fat and lean mass components, the associations of LMI or BF with baseline cardiovascular factors and cardiac remodelling are entirely different. Patients with higher LMI had a benign cardiovascular profile, lower MR degree and increased LV mass and LVEDV, while patients with higher BF had more concomitant clustered cardiovascular conditions and an increased LVOT gradient, MR degree and diastolic dysfunction. With respect to outcomes, reversed J-shape relationships of BMI and LMI with mortality were observed. Patients with higher BMI or LMI were related to a lower risk of mortality, especially in the low range of BMI and LMI. BF was not significantly associated with mortality in HCM patients.

## Data Availability

The original contributions presented in the study are included in the article/**Supplementary Material**, further inquiries can be directed to the corresponding author.

## References

[1] FinocchiaroGMagavernESinagraGAshleyEPapadakisMTome-EstebanM Impact of demographic features, lifestyle, and comorbidities on the clinical expression of hypertrophic cardiomyopathy. J Am Heart Assoc. (2017) 6(12):e007161. 10.1161/JAHA.117.00716129237589PMC5779031

[2] HorwichTBFonarowGCClarkAL. Obesity and the obesity paradox in heart failure. Prog Cardiovasc Dis. (2018) 61(2):151–6. 10.1016/j.pcad.2018.05.00529852198

[3] SpeltaFFratta PasiniAMCazzolettiLFerrariM. Body weight and mortality in COPD: focus on the obesity paradox. Eat Weight Disord. (2018) 23(1):15–22. 10.1007/s40519-017-0456-z29110280

[4] ForlivesiSCappellariMBonettiB. Obesity paradox and stroke: a narrative review. Eat Weight Disord. (2021) 26(2):417–23. 10.1007/s40519-020-00876-w32124408

[5] RobertsonJSchaufelbergerMLindgrenMAdielsMSchiölerLTorénK Higher body mass Index in adolescence predicts cardiomyopathy risk in midlife. Circulation. (2019) 140:117–25. 10.1161/CIRCULATIONAHA.118.03913231132859PMC6635044

[6] OreopoulosAEzekowitzJAMcAlisterFAKalantar-ZadehKFonarowGCNorrisCM Association between direct measures of body composition and prognostic factors in chronic heart failure. Mayo Clin Proc. (2010) 85:609–17. 10.4065/mcp.2010.010320592169PMC2894716

[7] PengYChenFHuangFYXiaTLHuangBTChaiH Body composition and mortality in coronary artery disease with mild renal insufficiency in Chinese patients. J Ren Nutr. (2017) 27:187–93. 10.1053/j.jrn.2017.01.01828320575

[8] CheitlinMDArmstrongWFAurigemmaGPBellerGABiermanFZDavisJL ACC/AHA/ASE 2003 guideline update for the clinical application of echocardiography: summary article: a report of the American college of cardiology/American heart association task force on practice guidelines (ACC/AHA/ASE committee to update the 1997 guidelines for the clinical application of echocardiography). Circulation. (2003) 108:1146–62. 10.1161/01.CIR.0000073597.57414.A912952829

[9] MaronBJ. Hypertrophic cardiomyopathy: a systematic review. JAMA. (2002) 287:1308–20. 10.1001/jama.287.10.130811886323

[10] MaronMSOlivottoIBetocchiSCaseySALesserJRLosiMA Effect of left ventricular outflow tract obstruction on clinical outcome in hypertrophic cardiomyopathy. N Engl J Med. (2003) 348:295–303. 10.1056/NEJMoa02133212540642

[11] PanzaJAPetroneRKFananapazirLMaronBJ Utility of continuous wave Doppler echocardiography in the noninvasive assessment of left ventricular outflow tract pressure gradient in patients with hypertrophic cardiomyopathy. J Am Coll Cardiol. (1992) 19:91–9. 10.1016/0735-1097(92)90057-T1729351

[12] LancellottiPMouraLPierardLAAgricolaEPopescuBATribouilloyC European Association of echocardiography recommendations for the assessment of valvular regurgitation. Part 2: mitral and tricuspid regurgitation (native valve disease). Eur J Echocardiogr. (2010) 11:307–32. 10.1093/ejechocard/jeq03120435783

[13] HuangFYWangHHuangBTLiuWPengYZhangC The influence of body composition on the N-terminal pro-B-type natriuretic peptide level and its prognostic performance in patients with acute coronary syndrome: a cohort study. Cardiovasc Diabetol. (2016) 15:58. 10.1186/s12933-016-0370-027048159PMC4822263

[14] Gomez-AmbrosiJSilvaCGalofreJCEscaladaJSantosSMillánD Body mass index classification misses subjects with increased cardiometabolic risk factors related to elevated adiposity. Int J Obes (Lond). (2012) 36:286–94. 10.1038/ijo.2011.10021587201

[15] LavieCJDe SchutterAPatelDARomero-CorralAArthamSMMilaniRV Body composition and survival in stable coronary heart disease: impact of lean mass index and body fat in the “obesity paradox”. J Am Coll Cardiol. (2012) 60:1374–80. 10.1016/j.jacc.2012.05.03722958953

[16] O'MahonyCJichiFPavlouMMonserratLAnastasakisARapezziC A novel clinical risk prediction model for sudden cardiac death in hypertrophic cardiomyopathy (HCM risk-SCD). Eur Heart J. (2014) 35:2010–20. 10.1093/eurheartj/eht43924126876

[17] GrambschPMTherneauTM. Proportional hazards tests and diagnostics based on weighted residuals. Biometrika. (1994) 81:515–26. 10.1093/biomet/81.3.515

[18] OlivottoIMaronBJTomberliBAppelbaumESaltonCHaasTS Obesity and its association to phenotype and clinical course in hypertrophic cardiomyopathy. J Am Coll Cardiol. (2013) 62:449–57. 10.1016/j.jacc.2013.03.06223643593

[19] ToczylowskiKHirnleTHarasiukDZabielskiPLewczukADmitrukI Plasma concentration and expression of adipokines in epicardial and subcutaneous adipose tissue are associated with impaired left ventricular filling pattern. J Transl Med. (2019) 17:310. 10.1186/s12967-019-2060-731533725PMC6751580

[20] PresslerAHallerBScherrJHeitkampDEsefeldKBoscheriA Association of body composition and left ventricular dimensions in elite athletes. Eur J Prev Cardiol. (2012) 19:1194–204. 10.1177/174182671142245521885466

[21] AlpertMAOmranJMehraAArdhanariS Impact of obesity and weight loss on cardiac performance and morphology in adults. Prog Cardiovasc Dis. (2014) 56:391–400. 10.1016/j.pcad.2013.09.00324438730

[22] MiyajiYIwanagaYNakamuraTYasudaMKawamuraTMiyazakiS Interrelationship between the myocardial mass, fibrosis, BNP, and clinical outcomes in hypertrophic cardiomyopathy. Intern Med. (2016) 55:1261–8. 10.2169/internalmedicine.55.648027181530

[23] HanSSKimKWKimKINaKYChaeDWKimS Lean mass index: a better predictor of mortality than body mass index in elderly asians. J Am Geriatr Soc. (2010) 58:312–7. 10.1111/j.1532-5415.2009.02672.x20070416

[24] KokkinosPFaselisCMyersJPittarasASuiXZhangJ Cardiorespiratory fitness and the paradoxical BMI-mortality risk association in male veterans. Mayo Clin Proc. (2014) 89:754–62. 10.1016/j.mayocp.2014.01.02924943694

